The article "Recent trends in the use of bacteriophages as replacement of antimicrobials against food-animal pathogens" was retracted in 2025. Reasons: unreliable results or conclusions; concerns about the results or conclusions; concerns about the article.

# Recent trends in the use of bacteriophages as replacement of antimicrobials against food-animal pathogens

**DOI:** 10.3389/fvets.2023.1162465

**Published:** 2023-05-25

**Authors:** Sana Zia, Khalid A. Alkheraije

**Affiliations:** ^1^Department of Zoology, Government Sadiq College Women University Bahawalpur, Bahawalpur, Pakistan; ^2^Department of Veterinary Medicine College of Agriculture and Veterinary Medicine, Qassim University, Buraidah, Saudi Arabia

**Keywords:** antimicrobials resistance, food security, bacteriophages, public health, food-animal pathogens, quality of life, pathogenesis

## Abstract

A major public health impact is associated with foodborne illnesses around the globe. Additionally, bacteria are becoming more resistant to antibiotics, which pose a global threat. Currently, many scientific efforts have been made to develop and implement new technologies to combat bacteria considering the increasing emergence of multidrug-resistant bacteria. In recent years, there has been considerable interest in using phages as biocontrol agents for foodborne pathogens in animals used for food production and in food products themselves. Foodborne outbreaks persist, globally, in many foods, some of which lack adequate methods to control any pathogenic contamination (like fresh produce). This interest may be attributed both to consumers’ desire for more natural food and to the fact that foodborne outbreaks continue to occur in many foods. Poultry is the most common animal to be treated with phage therapy to control foodborne pathogens. A large number of foodborne illnesses worldwide are caused by *Salmonella* spp. and *Campylobacter*, which are found in poultry and egg products. Conventional bacteriophage-based therapy can prevent and control humans and animals from various infectious diseases. In this context, describing bacteriophage therapy based on bacterial cells may offer a breakthrough for treating bacterial infections. Large-scale production of pheasants may be economically challenging to meet the needs of the poultry market. It is also possible to produce bacteriophage therapy on a large scale at a reduced cost. Recently, they have provided an ideal platform for designing and producing immune-inducing phages. Emerging foodborne pathogens will likely be targeted by new phage products in the future. In this review article, we will mainly focus on the Bacteriophages (phages) that have been proposed as an alternative strategy to antibiotics for food animal pathogens and their use for public health and food safety.

## 1. Introduction

Food safety is always a topmost priority in terms of public health and becomes more significant while considering animal-origin protein including eggs and meat. Many food-borne pathogens can cause illness in poultry birds starting from the initial hatch to the meal preparations (1). Antibiotics are used in the livestock and poultry industry for a century to treat diseases, parasites, and animals, promote growth at subtherapeutic doses in animal feed, and improve animal products (2). Antibiotics are highly efficient against bacterial infections, saving millions of lives and drastically reducing mortality rates. However, multidrug-resistant bacteria (MDR), extensively drug-resistant bacteria (XDR), and even pan-resistant bacteria (PDR) have evolved because of antibiotic overuse, abuse, and misuse. Antibiotics are currently ineffective against infections caused by drug-resistant bacteria (3). As the antibiotic drug discovery pipeline is failing, finding new drugs is becoming increasingly critical. Consumer awareness about preservation in a chemical way in the food and on processing surfaces has also led to an increase in interest in natural antimicrobial agents (4). They can boom in a wide variety as pathogens emerge all through treatment, have the simplest minor results on regular flora, are similarly powerful against antibiotic-resistant bacteria, are without problems detected, break bacterial biofilms, and are often non-toxic (5).

The article "Recent trends in the use of bacteriophages as replacement of antimicrobials against food-animal pathogens" was retracted in 2025. Reasons: unreliable results or conclusions; concerns about the results or conclusions; concerns about the article.

A variety of pathogens have been found in soil, ground and surface water, food (e.g., sauerkraut and wine), sewage, and sludge (6). In addition to humans and animals, they have also been isolated from feces, urine, saliva, spit, rumens, and serum (7). With their bacterial hosts, phages are part of the intestinal flora because of their ability to penetrate different organs and tissues (8). The trophic effect of these bacteria limits bacterial populations in aquatic ecosystems by 10 to 80% (9). In terms of their morphology and size, bacteriophages are classified into different families. The majority of them have tails, but they also have filaments and pleomorphic (10). There are two basic components of a phage virion: nucleic acid (dual- or single-stranded RNA or DNA) and a protein envelope. Lipids are sometimes part of the envelope or of the lipid wall (11). In the course of bacteriophages’ occurrence, viability, and storage, various external physical and chemical factors, including temperature, acidity, salinity, and ions, play a significant role. Damage to a phage’s structural elements, loss of lipids, and/or changes in DNA structure can inactivate a phage (12).

In recent years, there has been a lot of interest in using phages to control pathogens (13). Studies have examined the use of phages as indicators of fecal contamination and as antimicrobials (14). They are currently one of the promising antibiotic alternatives with the most potential because of their ability to effectively combat bacterial infections. Phages are a new alternative therapy under the “one health” approach that can be used to control bacteria in plants, animals, food, and humans and they are very common in all natural environments and play an important role in bacterial evolution (15). Phages can be categorized into two types, namely virulent (exclusively undergo the lytic cycle) and temperate (are able to endure the lysogenic cycle). Phages are very specific as each type generally attacks different bacterial species. Virulent phages enter the bacterial cell, replicate using the host machinery and finally lyse the host cell, leading to the disintegration of the bacteria (16). Viral phages replicate much faster than host bacteria when they infect a bacterium. Within 30–40 min, the entire cycle can be completed. Phages are parasites that propagate by taking advantage of their hosts, which can be affected by temperature, nutrient levels, and various environmental factors (17). The purpose of this review is to discuss various issues that are related to antibiotic resistance as well as the use of bacteriophages as a cure against antimicrobial resistance against food-animal pathogens.

The article "Recent trends in the use of bacteriophages as replacement of antimicrobials against food-animal pathogens" was retracted in 2025. Reasons: unreliable results or conclusions; concerns about the results or conclusions; concerns about the article.

## 2. Recent antimicrobial resistance status in food animal pathogens

Antimicrobial resistance is a serious public health issue that poses a grave threat to the spread of incurable infections. Many emerging infectious diseases around the world are now caused by antibiotic-resistant bacteria (18). Although antimicrobial resistance is a natural result of how microbes evolve, human production abuse of antimicrobial drugs has accelerated resistance to transfer in a variety of pathogenic and microbiome pathogens (19). Even medical and public health professionals understand the significance of antimicrobial use in agriculture as a component of antimicrobial resistance (20). It is well known that antibiotic resistance is one of the most significant issues affecting bacterial pathogens around the world (21). Infections caused by Gram-positive and Gram-negative bacteria have developed multidrug resistance patterns that make conventional antimicrobials ineffective or even untreatable. There is a lack of early identification of causative microorganisms and antimicrobial susceptibility patterns in many healthcare settings, so wide-spectrum antibiotics are routinely and largely unnecessarily administered to patients with bacteremia and other serious infections (21). As a result of poor infection control practices and escalating resistance rates, bacteria can spread rapidly from patient to patient and into the environment. A practical antimicrobial stewardship program in hospitals can be developed when updated epidemiological data are available on antimicrobial resistance in frequently encountered bacterial pathogens (21). There is an alarming rise in multidrug-resistant bacteria and resistance to common antimicrobial therapies. Bacterial infections and their associated diseases pose a challenge, and since there are currently fewer effective drugs, fewer effective prevention measures, and only a few new antibiotics in clinical trials, novel treatment options, and alternative antimicrobial therapies are required (22).

The article "Recent trends in the use of bacteriophages as replacement of antimicrobials against food-animal pathogens" was retracted in 2025. Reasons: unreliable results or conclusions; concerns about the results or conclusions; concerns about the article.

The intensity of antimicrobial use in agriculture is insufficient and dwarfs the scale of clinical use and misuse, even though clinical concerns are not trivial. Additionally, the growing issue of drug-resistant food-borne infections is rarely linked to the production of food animals, which reduces the efficacy of public health initiatives to prevent food-borne illness (23). Most signification, rather than conceptualizing issues ecologically in terms of resistance gene reservoirs that may spread throughout the microbial ecosystem, the problem is frequently conceptualized in terms of resistance to specific antimicrobials in clinically important pathogens (24). As agricultural antibiotic use changed, researchers tracked the prevalence of antimicrobial resistance in ecological studies. Research on cross-sectional groups is considered to be cross-sectional if it focuses on specific groups that are in close contact with antimicrobial-treated food animals or farming families (e.g., farmers) (25). Bacteria that are resistant to antibiotics can be found in the home, animal waste, and the environment. Thirdly, researchers examined antibiotic resistance in bacteria isolated from conventional producers and those who did not use antibiotics (26).

## 3. Mechanism of bacteriophages

There are billions of viruses on the planet. The number of viruses in the universe is estimated to be 1,031, which is far greater than the number of stars (27). As part of the viral population, bacteria are infected and devoured by bacteriophages, or phages. Phyto phages are unique in their potential antibacterial properties (28). There are many phages in every ecosystem, and they are considered the most abundant and diverse organisms on the planet (29). In addition to hunting for a specific bacterium species, phage particles can hunt for a subset of the same species. Phages replicate inside bacteria after they infect them. Phages multiply exponentially after infecting a bacterial cell, taking advantage of the bacteria’s protein synthesis and energy-producing machinery. The protein synthesis and energy-producing machinery of bacteria are used by phages to multiply exponentially after infecting a bacterial cell. Nevertheless, lysis and lysogenesis are two ways of propagating bacteria. In the case of lytic phages, the bacterial cell is lysed before the virus is released (30). A lysogenic phage integrates its genome into the bacterium that replicates it and acquires new characteristics for the bacteria. It shows that phage is important for treating both local and systemic infections in humans (31). It is worth noting that the development of antibiotic resistance in bacteria has not kept the development of different stages of resistance in bacteria, instead, the fact that phage resistance may be a significant issue in bacteria. More therapy of phage has been shown to be safe and relatively free of side effects (32). In antimicrobial phage therapy, bacteriophages are used because they can recognize, adsorb, multiply, and cause lysis of bacteria only inside their cells (33). In its most basic form, phage therapy refers to the use of infectious bacteria-specific viruses to inhibit the growth of pathogenic bacteria (34). In most cases, bacteriophage may be effective against Gram-positive and negative bacteria that are resistant to antibiotics (35).

The article "Recent trends in the use of bacteriophages as replacement of antimicrobials against food-animal pathogens" was retracted in 2025. Reasons: unreliable results or conclusions; concerns about the results or conclusions; concerns about the article.

### 3.1. Lytic phage

For the lytic cycle to begin, the phage must attach to the bacterium using a protein (13). The genetic material of the bacteriophage is incorporated into the bacterial host cell after the attachment of the viral particle. Phages use bacterial metabolic machinery to make copies of DNA or RNA from their genetic material upon entry (36). DNA viruses copy themselves directly into messenger RNA (mRNA) molecules that are used to control the host’s ribosomes. Retroviruses (RNA viruses) are transcribed into DNA by reverse transcriptase, which then follows the pathway followed by the DNA virus to transcribe viral RNA. In the later stages of the translation, the newly translated proteins are assembled to form the capsid and tail of the phages, which are released from the host cell. Infecting and multiplying new host cells are the next steps for the newly formed particles. During phage replication, the host chromosome is sometimes packed into the capsid instead of the phage genome, representing an example of horizontal gene transfer (37). Direct applications of lytic-cycle-only phages include addressing antibiotic-resistant pathogenic bacteria using their appropriate lytic cycles.

### 3.2. Lysogenic phage

A lysogenic cycle characterized by the integration of viral genetic fabric into the bacterial genome (referred to as a prophage) and persevered replication of viral genetic cloth without deadly outcomes for the inflamed host (38), is particularly prevalent in temperate phages. Infection with viral genetic material can change the bacteria’s phenotype, however, because the virus incorporates genetic material into the host. It is evident that many common bacterial strains are pathogenic as a result of this conversion. Hydrogen peroxide can also be used to prevent such lysogenic conversion by producing reactive oxygen species, glutathione, and overexpressing transcriptional repressors (39).

The article "Recent trends in the use of bacteriophages as replacement of antimicrobials against food-animal pathogens" was retracted in 2025. Reasons: unreliable results or conclusions; concerns about the results or conclusions; concerns about the article.

## 4. Bacteriophages against food animal pathogens-mechanisms and *in-vitro* studies

*Escherichia coli, Campylobacter, Salmonella*, and *Listeria* are the four most common foodborne pathogens of animal origin (40). Most of the time, these bacteria are carried asymptomatically in the gastrointestinal tracts of ruminants, poultry, and swine. To prevent animal disease and/or reduce gastrointestinal pathogen transport, which prevents pathogen entry into the food supply, phage administration to cattle is used as a direct pre-harvest strategy. The application of phages directly to animal carcasses is the basis of post-harvest strategies, aimed at cleaning the product (41).

### 4.1. Escherichia coli

The bacterium *E. coli* is Gram-negative. Food poisoning is frequently caused by *E. coli*, particularly the serotype O157:H7 strain, which produces the Shiga toxin (42). Its primary reservoir is ruminants, and because it thrives in intestinal environments, improper handling during slaughter may result in the contamination of meat with feces, dust from the hide, or intestinal contents. *E. coli* is most transmitted to humans through raw contaminated food, and raw milk and water are thought to be associated with cases of cross-contamination involving direct or indirect contact with feces. These microbes are highly toxic and a public health hazard because they can spread infections when ingested in concentrations as low as 10 cells (43). The application of phages to poultry has been successful to prevent fatal respiratory infections in broiler chickens (44). Several different approaches have been used; however, aerosol spraying and intramuscular (a.m.) injection have given the best results and reduced significantly the mortality of broiler chicken. Despite these results, phage administration in addition to bird drinking water proved to be inefficient in protecting the birds from fatal *E. coli* respiratory infections (45). The main speculated causes for the failure of oral treatments have been reported to be (i) nonspecific binding of phages to food particles and other debris in the rumen and gastrointestinal tract (46); (ii) phage inactivation upon contact with the acidic conditions of the abomasum (iii) causing an insufficient number of oral phages reaching the gastrointestinal tract. An interesting approach to reducing coliphage inactivation has been described by Stanford and colleagues in 2010. These authors successfully encapsulated phages in polymeric matrices which resisted *in vitro* acidic conditions and furthermore, once delivered orally to steers caused the reduction of *E. coli* levels (47) (Table 1).

The article "Recent trends in the use of bacteriophages as replacement of antimicrobials against food-animal pathogens" was retracted in 2025. Reasons: unreliable results or conclusions; concerns about the results or conclusions; concerns about the article.

**Table 1:** Pre-and post-harvest use of *E. coli, Campylobacter, Salmonella*, and *Staphylococcus aureus* phage.

Animal	Plan	Phage	References
**Postharvest application**			
Meat	Applied on top	e11/2, e4/1c, pp01	(48)
Current produce (lettuce, cantaloupe)	Sprayed	Bacteria cocktail (ECP-100)	(49)
Food is exposed (spinach blades)	Sprayed	Bacteria cocktail	(50)
Food is exposed (steel, ceramic chips)	Applied on top	BEC8	(51)
Chicken	Put on top	Φ2	(52)
Chicken skin	Put on top	Φ29C	(53)
Meat (Beef)	Cj6	Cj6	(54)
Foods that are ready to eat and chocolate milk	Milk is mixed in and added to foods.	FO1-E2	(55)
Meat (pig)	Bacteria cocktail (PC1)	Phage cocktail (PC1)	(55)
Meat (raw/cooked beef)	Applied on top	P7	(56)
Meat (Skin chicken)	Applied on top	P22, 29C	(57)
Prepared meals (cheese)	Included in the pasteurized milk vat	vB_SauS-phi-IPLA35, vB_SauS-phi-SauS-IPLA88	(58)
Prepared food (milk curd)	To whole milk that has been pasteurized	Cocktail (Φ88 and Φ35)	(58)
Raw dairy products like whey	Added to raw milk whey	K	(59)
ready-to-eat foods that are raw (milk products and derivatives)	Add to milk	K	(59)
**Preharvest application**			
Ruminant (sheep)	Oral delivery	CEV1, CEV2	(60)
Ruminant (cattle)	Oral delivery	e11/2, e4/1c	(61)
Ruminant (cattle)	Oral/rectal delivery (via drinking water)	KH1, SH1	(62)
Poultry (broiler chicken)	Injection into the left thigh	SPR02 and DAF6	(52)
Poultry (Chickens broiler)	oral transmission (oral gavage and in feed)	Phage cocktail	(52)
Poultry (Broiler chickens)	Poultry (Broiler chickens)	69, 71	(63)
Swine (Weaned pigs)	Oral delivery	Phage cocktail	(64)
Chickens	Oral delivery	Phage cocktail (CB4ϕ, WT45ϕ)	(65)
Poultry	Antacid suspension	Φ151, Φ25, Φ10	(56)
Pig	Oral delivery	Felix01	(66)

### 4.2. Campylobacter

The ideal growth temperature for Gram-negative, spiral, motile, and microaerophilic bacteria belonging to the genus *Campylobacter* is 41°C (61). Members of *C. jejuni* and *E. coli* are considered the main etiological agents of enteric diseases worldwide. Due to the possibility of campylobacteriosis, which is usually characterized by fever, bloody diarrhea, and excruciating abdominal pain, when low doses (400–500 cells) are administered, this widespread infection has been described (52). Because Campylobacter can colonize the intestines of chickens and cattle, infection usually occurs through mouth-to-mouth contact, consumption of contaminated food (such as raw meat and milk that has been contaminated with feces), and contaminated drinking water. Spread by water. Several strategies to control this infection using bacteriophages have been developed because of the disease’s widespread occurrence and financial impact on the agriculture and food industries (67). It is known that *Campylobacter* attaches and forms biofilms on surfaces as a measure to overcome environmental stresses, such as aerobic conditions, desiccation, heating, disinfectants, and acidic conditions frequently encountered in food environments (36); however, data, we were only able to find one report evaluating the efficacy of Campylobacter phages of disrupting biofilm formed on the glass. In this study, phages were able to reduce by 1 to 3 log the viable cell counts under microaerobic conditions; however, after treatment above 84% of the surviving bacteria were resistant to the two phages applied (68).

The article "Recent trends in the use of bacteriophages as replacement of antimicrobials against food-animal pathogens" was retracted in 2025. Reasons: unreliable results or conclusions; concerns about the results or conclusions; concerns about the article.

### 4.3. Salmonella

A genus of facultative intracellular species that are Gram-negative known as *Salmonella* is believed to account for a significant proportion of zoonotic diseases reported worldwide. It is frequently linked to consuming tainted food of animal origin because *Salmonella* serovars have the ability to colonize and survive in the human gastrointestinal tract (55). Each year, *Salmonella* infections cost the Europe Union (EU) healthcare system around three million euros. Most *Salmonella* outbreaks are attributed to the consumption of tainted meat and eggs from poultry, pork, and cattle, respectively. *Salmonella* is another bacterium that can spoil processed foods. This microorganism, when ingested, can cause diseases, fever, diarrhea, and pain (40). Unlike phage preharvest strategies on animals, several postharvest strategies have adopted the use of only one phage and not a cocktail. All *Salmonella* phages reported have been able to decrease the number of viable cells present in raw meats, D processed and ready-to-eat foods, and fresh produce (69). Furthermore, the combined treatment of phage and *Enterobacter asburiae*, a strain exhibiting antagonistic activity against *Salmonella*, to control this pathogen on tomatoes, mung bean sprouts, and alfalfa seeds, represents a highly promising, chemical-free approach. However, in some settings phages were found to be readily immobilized by the food matrix and, although retaining infectivity, they lost the ability to diffuse and infect target cells (55).

The article "Recent trends in the use of bacteriophages as replacement of antimicrobials against food-animal pathogens" was retracted in 2025. Reasons: unreliable results or conclusions; concerns about the results or conclusions; concerns about the article.

### 4.4. Staphylococcus aureus

Gram-positive *S. aureus* is a typical way for mastitis in dairy cows and is considered a serious threat to food safety. According to the Central Depository Company (CDC), there are 242,148 cases of staphylococcal food poisoning in the United States annually. Eating foods that have an adequate amount of one or more enterotoxins in them causes this condition (59). *S. aureus* contamination of food has been linked to a variety of mechanisms, including human handling of food products, livestock infection and colonization, and human infection and handling of farm animals. Although most people recover in 1–3 days after experiencing mild symptoms, *S. aureus* can cause poisoning within 1 to 6 h after consuming contaminated food. It is estimated that mastitis in adult dairy cows causes losses of US$ 35 billion per year. Dairy food products and the majority of lactating cows have been the focus of phage research (70).

### 4.5. Clostridium

*Clostridium perfringens* is spore-forming rods, non-motile and Gram-positive which are normally found in poultry’s intestinal microbiota. As low as 10^4^ CFU are present, it is not pathogenic, but its pathogenicity is primarily due to its toxins. Necrotic enteritis (NE) occurs both in acute clinical and subclinical forms in chickens and is one of the most economically important diseases of poultry caused by *Clostridium perfringens* type A and type C-producing toxins. Additionally, infected poultry meat may cause human illness when it is infected with *C. perfringens* produces enterotoxins (71). Bacteriophages derived from *C. perfringens* strains isolated from poultry intestines and soils, as well as those isolated from soils and sewage, were identified as *Siphoviridae* and *Podoviridae* bacteria. Despite the phages, many strains of *C. perfringens* remained resistant to them. Specific isolation of this bacterium was also shown to be resistant to the activity of phages. *C. perfringens* phages encode endolysin, which may be particularly useful for controlling this bacterium, according to some authors. Despite differences in sensitivities between strains of *C. perfringens*, the results indicate that endolysin is active against all strains tested (62, 72). reported a decreased incidence of necrotic enteritis (NE) in broiler chickens after bacteriophage (INT-401) treatment. Experimentally infected broiler chickens also gained more weight and had a better feed conversion ratio with phage treatment *via* drinking water or feed.

## 5. Field and lab animal trials of bacteriophages in infectious diseases of food animals

The most popular model in studies on phage therapy is poultry. It was found to be very successful to combine two bacteriophages that are lytic for *Campylobacter jejuni*. The experiment was conducted on first-caught, 25-day-old broiler chickens. Broilers were kept separate from Jejuni. It was found that the type and dosage of bacteriophages used had an impact on phage therapy’s efficacy (34). According to Wagenaar et al. (73), prophylactic oral administration of a mixture of phages (phage strains 69 and 71) to chickens delayed colonization of the gastrointestinal tract by *C. jejuni* and resulted in this level of colonization within 1 week. As viewed, stabilized. 2.0 in the treatment group following a first log reduction. Contrarily, after several days of phage therapy, *C. jejuni* counts had initially decreased by 3.0 logs, but they had only increased by 1 log compared to the untreated control group of chickens was lower (74). *E. coli* infection is a common problem for sheep farmers. Bacteriophages and their potential applications in the defense of sheep against *E. coli* infection were described by Bach et al. (75) Experimental sheep were exposed to four different strains of *E. coli* on day 0. On days 2, 1, 0, 6, and 7 of the trial, three bacteriophage cocktails (1,010 PFU of P5, P8, and P11 each) were administered orally. When stool samples were taken, the amount of *E. coli* was reduced (75). Mice are yet another common model used in phage therapy research. *Salmonella enterica* serotype enteritidis infection control in mice using phage treatment. Five-week-old female BALB/c mice with a mean weight of 20 g were obtained and weighed in order to assess the impact of phage SE20 on salmonellosis (76). The salmonellosis model and animal testing were done. Twenty-four mice were divided into three groups; in group A, which served as the control, 200 L of PBS was gavage; in group B, 200 L of *S. enteritidis* (1.5 × 107 CFU/mL) was gavage; and in group C, 200 L of *S. enteritidis* (1.5 × 107 CFU/mL) was gavage on the first day, and a single dose of phage SE20 was gavage. Anti-acid was gavage into the animal’s stomach to protect the phages there from harm. After six days of infection, four mice from each group were put to sleep. Histopathology of the liver and spleen. The liver and spleen were then taken out and preserved in 10% formalin for 24 h at 6°C in the refrigerator (76).

The article "Recent trends in the use of bacteriophages as replacement of antimicrobials against food-animal pathogens" was retracted in 2025. Reasons: unreliable results or conclusions; concerns about the results or conclusions; concerns about the article.

## 6. Bacteriophages products available in market

A growing number of businesses worldwide are developing and commercializing phage biocontrol products because of the biological properties of lytic bacteriophages. Phage biocontrol, however, has some drawbacks and restrictions (77). Over the past 12 years, the number of regulatory approvals granted for the use of bacteriophage preparations to improve food safety has steadily increased (Table 2). The Food and Drug Administration (FDA) approved - *L. monocytogenes*-specific cocktail ListShieldTM as a food enhancer in 2006 as the first bacteriophage preparation for direct use in food (the FDA labels any product as “not approved” alternatively, the term “approval” is often used to indicating that obtaining FDA clearance means using the products for their intended applications) (81). Later that year, the FDA approved Listex TM (now Phage Guard Listex TM), Listeria guidelines, as a Generally Recognized as Safe (GRAS) substance. The FDA recently granted GRAS status to several phage products, including SalmoFreshTM and Phage Guard STM. As a result, applying for GRAS status now seems to be the standard for phage products for post-harvest food processing. Since wild-type (i.e., not genetically modified) soluble bacteriophages are completely natural and already present in food, the GRAS designation seems to be an appropriate regulatory pathway for these agents. Phage preparations can be used in the production of meat, poultry, and egg products. It is legal to use phages on food (e.g. *Salmonella* targeting phage) and livestock prior to slaughter (82). USDA has included information on several phage preparations in its published guidelines. Although these directives are made using specific phage preparations, in general, any phage product that meets the requirements of the directives may be considered legal. Several health organizations around the world have approved the use of phage products in food, following the example of US regulators (79, 80).

**Table 2:** Types of bacteriophage products available in the market.

Agency name	Product	Bacteria	References
Intralytix Inc.	ListShield™	*L. monocytogenes*	(78)
FINK TEC GMBH	EcoShield™	*E. coli*	(79, 80)
Intralytix, Inc.	SalmoFresh™	*Salmonella* spp.	(81)
Micreos Food Safety	Phage Guard S™	*Salmonella* spp.	(82)
Micreos Food Safety	Phage Guard Listex™	*L. monocytogenes*	(83)
Intralytix, Inc.	Shiga Shield™ (ShigActive™)	*Shigella* spp.	(84)
Phagelux	Agri Phage™	*Xanthomonas campestris* pv. Vesicatoria *Pseudomonas syringae* pv. tomato	(83)
Phagelux	SalmoPro®	*Salmonella* spp.	(82)
Passport Food Safety Solutions	Finalyse®	*E. coli*	(85)

Phage products are non-genetically modified organisms (non-GMO), GMO-free phages that stay in a solution that is biocontrol chemicals. In comparison to other safety intervention techniques, these phage products are inexpensive, costing only per pound of treated food. These commercially available phage products are regarded as eco-friendly and organic sciences (78). Phage products such as these typically contain naturally occurring, GMO-free phages suspended without harsh chemicals commonly used in biocontrol. A phage product costs between 1–4 cents per pound of treated food, compared to other safety intervention techniques that typically cost between 10 and 30 cents per pound. The dramatic price difference between phage biocontrol products and existing interventions is another major advantage (83). It is essential to keep in mind that this represents the cost of a constructed item to treat a single pathogen. Using multiple products increases the overall cost of phage biological control. More and more companies are developing and marketing phage biocontrol methods that will increase their usefulness in the food industry (86).

The article "Recent trends in the use of bacteriophages as replacement of antimicrobials against food-animal pathogens" was retracted in 2025. Reasons: unreliable results or conclusions; concerns about the results or conclusions; concerns about the article.

## 7. Economic impacts of the use of bacteriophages

A major problem in food production facilities development such as microbiological bacilli on equipment surfaces. Bacterial biofilms are defined as aggregates of cells attached to biotic or abiotic surfaces and enclosed in an extracellular polymeric matrix consisting of self-assembly (EPS) (23). Biofilm-forming bacteria have a high level of resistance to harmful environmental factors, antibiotics, and cleaning agents. The majority of pathogenic bacteria in the fresh produce industry, including *L. monocytogenes, Salmonella, E. coli, and Yersinia,* can attach to plant tissues where they can grow and form biofilms. Because of the inherent structure of vegetables, these microorganisms have a harder time accessing sanitizers (87). In order to remove the biofilm on plant tissues, preparations that are safe for humans must be developed. Bacteriophages offer hope for developing human-safe sanitizers (88). *Campylobacter jejuni* is one of the pathogenic bacteria that can form biofilms on materials frequently used in industries (i.e. polyvinyl chloride and stainless steel). On glass Petri plates, *C. jejuni* biofilm formation was prevented using the lytic bacteriophages CP8 and CP30 that were isolated from chicken excrement (89). In comparison to a control biofilm that had not been treated with bacteriophage, The viable count was found to be reduced by 1.0–3.0 log CFU/cm2 24 h after infection following phage treatment of each biofilm, according to the research depending on the strain that forms a biofilm, there were differences in the degree of reduction and the potential for phage resistance (90). When compared to *C. jejuni* strain NCTC 11168, *C. jejuni* strain PT14 was distinguished by its ability to produce a much larger amount of biofilm on glass. No resistant *C. jejuni* cells were found in the PT14 biofilm treated by phages among the bacteria that made it through the bacteriophage treatment. Eighty-four percent of the *C. jejuni* 11,168 cells showed resistance to phage CP8 and 90 % showed resistance to phage CP30 (91). No resistant *C. jejuni* cells were found in the PT14 biofilm treated by phages among the bacteria that made it through the bacteriophage treatment. Eighty-four percent of the *C. jejuni* 11,168 cells showed resistance to phage CP8 and 90% showed resistance to phage CP30 (68). Endolysins are an enzyme made by bacteriophages that may be used in sanitization. Bacteriophages produce endolysins at the end of their lytic cycle, which allows the release of progeny virions by breaking down peptidoglycan found in the cell wall. Gram-positive bacteria can also be exogenously injected with them to kill them; Gram-negative bacteria have an outer membrane that shields them from endolysin activity. Based on where they cleave the peptidoglycan, lysins are divided into five groups: glycosaminidases, lytic transglycosylases, muramidase, amidases, and endopeptidases (92). Staphylococcal counts in the polystyrene-adhered biofilm were found to be reduced by 1.0–3.0 log units by endolysin LysH5, a product of the *S. aureus* phage vB SauS-phiIPLA88. Oliveira et al. (93) claim that an additional factor that acts on the bacterial envelope is necessary to disestablish the outer membrane in order to achieve good efficacy with endolysins against bacteria. It has also demonstrated that LysK endolysin and DA7 depolymerase work together to inhibit staphylococcus biofilm. These two enzyme mixtures in nano- and micromolar concentrations can remove biofilm from polystyrene and glass surfaces even at very low concentrations (89).

The article "Recent trends in the use of bacteriophages as replacement of antimicrobials against food-animal pathogens" was retracted in 2025. Reasons: unreliable results or conclusions; concerns about the results or conclusions; concerns about the article.

## 8. Challenges to the use of bacteriophages

To cope with the emergence of multi- and pan-drug resistant bacterial lines, new antimicrobial agents and therapeutic techniques are wished. As we input the submit-antibiotic generation, bacteriophages are considered the most promising way to the cutting-edge scientific disaster, with several benefits over traditional antimicrobials. It is unusual that phage therapy (PT) has produced big progress over a long time, however, gaps need to still be recognized and filled, the phage-based preparations ought to be secure and powerful to be used in hen production, chicken medication, and the rooster enterprise. Further to the dosage and management technique (consisting of education of fashionable formulations), the timing of administration of phage-primarily based merchandize in addition to concomitant preparations (together with competitive exclusion) or vaccination is essential. Bacteriophages can survive longer on meat product surfaces when refrigerated. To achieve positive outcomes for human health and well-being, action must be taken, and methods and practices must be modified (94). Designed for use in the poultry industry, phage-based formulations must be safe and effective. In addition to dose and method of administration (including preparation of standardized formulations), staging of drugs, as well as the timing of concomitant drugs (e.g., competitive exclusion) or vaccination, is also important. Individual bacteriophages and environmental factors can affect the persistence of bacteriophages in food (e.g., temperature) (95).

The article "Recent trends in the use of bacteriophages as replacement of antimicrobials against food-animal pathogens" was retracted in 2025. Reasons: unreliable results or conclusions; concerns about the results or conclusions; concerns about the article.

The industry that produces food has to continuously contribute to attempts to stop infectious diseases and the problems with antibiotic resistance in human infections that come from food animals. Microbial safety issues continue to be a problem despite numerous technological advancements in methods for the detection and elimination of foodborne pathogens at each stage of the food production process, in good manufacturing practices, quality control and hygiene, changes in animal husbandry, and in agronomic procedures (96). There is a need for the development of alternative antibacterial approaches at the production level to maintain safety standards, control foodborne pathogens, and limit their detrimental effects on the food industry and on human health. In addition, the restricted use of some antibiotics during food animal production, coupled with the lack of development of new antimicrobials, has put additional strain on the food production sector (97). Bacteriophages (phages) are advantageous candidates for use in both the detection and control of pathogens at each stage of the food production process from farm to fork due to their natural specificity to infect and kill their target bacteria, as well as the fact that they are ubiquitous in the environment and harmless to humans and animals (98). To combat some of the most common foodborne pathogens, such *as Escherichia coli, Salmonella* serovars, and *Listeria monocytogenes*, a variety of phage-based products have recently entered the commercial market (99).

## 9. Prospects

Recent decades have seen an increase in phages being used as biocontrol tools as a result of AMR bacteria emerging and antibiotics being limited in use in livestock and crops (100). In the fight against bacteria, phages remain a fascinating and natural alternative As we discussed in previous sections, phages have numerous applications and advantages concerning food safety. There are some issues that must be resolved before these findings can be widely applied, despite their encouraging results (101). As well as being assets, phage specificity, resistance to resistance, and self-dosing capacity can also be liabilities. The phage specificity of these antimicrobials significantly limits their effectiveness in biocontrol. Bacterial capsules and cell walls contain receptors responsible for a majority of host tropism. When dealing with pathogenic bacteria, the task of building phage banks or biobanks can be stressful and time-consuming. In this situation, direct hunting is likely to be more efficient and cost-effective. In a fascinating development, biobanks may make phages readily available for lysing bacteria from various species. It is, however, necessary to perform programs to pick out the potential phages quickly (102, 103). Despite being rare, phage matching can be easily carried out with automated equipment, even though finding the precise phage can take some time. A phage biocontrol treatment can be successfully achieved as a customized treatment by hunting for phages, as well as knowing the bacterial host (88). Moreover, phages can be used as broad-range products when they are combined with broad-range phages. It may also be beneficial to broaden the host range by phage training (experimental evolution) or to develop chimeric phages able to recognize multiple strains or species, though this may negatively affect commensals. Food safety benefits from disinfectants that reduce bacterial burdens, and phage-derived enzymes, which can break down bacterial biofilms, may also offer promising solutions. It has been shown that phages produce hydrolytic proteins that are capable of actively destroying polysaccharide-based bacterial matrices and dislodging biofilms (88).

The article "Recent trends in the use of bacteriophages as replacement of antimicrobials against food-animal pathogens" was retracted in 2025. Reasons: unreliable results or conclusions; concerns about the results or conclusions; concerns about the article.

Another disadvantage is the inherently unstable nature of some phages. It may be necessary to take specific measures to keep phage-based products stable and, therefore, infective. To control phage release and deliver phages more precisely, nanoparticles can be embedded with phages. As a result of this method, commercial products may be stable over long periods and in a variety of environmental conditions (104). Besides freeze-drying, other preservation techniques might also be a viable option for long-term phage storage; they are significantly less expensive, making them an appealing choice for the industry. As phages lose their ability to maintain infectivity after processing, encapsulation may be the best method for protecting food (105, 106). It is also necessary to comply with legal requirements before using a phage application. It is, however, important to note that because of phages’ inherent evolvability, their diversity and morphologies, as well as their inherent evolution and ability to self-replicate in bacterial hosts, regulatory agencies face a challenge, highlighting the importance of applying the same regulations and procedures to all phage-derived products. As can be seen, phage regulation is a complex issue that will delay phage use for routine and commercial applications. The regulatory bodies should, however, propose phage biocontrol recommendations quickly as an alternative to antibiotics to combat the emergence of resistant bacteria (13).

The article "Recent trends in the use of bacteriophages as replacement of antimicrobials against food-animal pathogens" was retracted in 2025. Reasons: unreliable results or conclusions; concerns about the results or conclusions; concerns about the article.

## 10. Conclusion

Food safety and sustainability remain the most pressing global food industry challenges. The food manufacturing industry has continuously contributed to efforts to prevent infectious diseases and antibiotic resistance related to human pathogens from food animals. Several leading and emerging pathogens in food have been successfully controlled by bacteriophages, a class of natural antibacterial agents. Although bacteria phages (phages) are ubiquitous in the environment and harmless to humans and animals, they make excellent candidates for detecting and controlling pathogens from farm to fork. Their natural ability to infect and kill their target bacteria makes them a powerful tool for both detection and control. Food contamination can be managed by biological procedures such as bacteriophage biocontrol rather than using chemical preservatives as they become less available. For phage propagation, it is advantageous to select nonvirulent and genetically well-characterized bacteria. The establishment of safe large-scale production processes will be necessary for bacteriophages to be used as bio preservatives in the future. However, in food systems, phages’ antimicrobial activity could be greatly reduced as compared to laboratory conditions.

## Author contributions

SZ conceived the idea, wrote the original manuscript and KA revised the manuscript drew the figures and provide financial support.

## Conflict of interest

The authors declare that the research was conducted in the absence of any commercial or financial relationships that could be construed as a potential conflict of interest.

## Publisher’s note

All claims expressed in this article are solely those of the authors and do not necessarily represent those of their affiliated organizations, or those of the publisher, the editors and the reviewers. Any product that may be evaluated in this article, or claim that may be made by its manufacturer, is not guaranteed or endorsed by the publisher.
